# The Role of 3D Printing in Medical Applications: A State of the Art

**DOI:** 10.1155/2019/5340616

**Published:** 2019-03-21

**Authors:** Anna Aimar, Augusto Palermo, Bernardo Innocenti

**Affiliations:** ^1^Aid4Med S.r.l., Udine 33100, Italy; ^2^Head 3 Orthopaedic Department, Istituto Auxologico Italiano IRCCS Capitanio Hospital, Milan 20122, Italy; ^3^BEAMS Department, Université Libre de Bruxelles, Bruxelles 1050, Belgium

## Abstract

Three-dimensional (3D) printing refers to a number of manufacturing technologies that generate a physical model from digital information. Medical 3D printing was once an ambitious pipe dream. However, time and investment made it real. Nowadays, the 3D printing technology represents a big opportunity to help pharmaceutical and medical companies to create more specific drugs, enabling a rapid production of medical implants, and changing the way that doctors and surgeons plan procedures. Patient-specific 3D-printed anatomical models are becoming increasingly useful tools in today's practice of precision medicine and for personalized treatments. In the future, 3D-printed implantable organs will probably be available, reducing the waiting lists and increasing the number of lives saved. Additive manufacturing for healthcare is still very much a work in progress, but it is already applied in many different ways in medical field that, already reeling under immense pressure with regards to optimal performance and reduced costs, will stand to gain unprecedented benefits from this good-as-gold technology. The goal of this analysis is to demonstrate by a deep research of the 3D-printing applications in medical field the usefulness and drawbacks and how powerful technology it is.

## 1. Introduction

Among the different manufacturing processes that are currently adopted by the industry, the 3D printing is an additive technique. It is a process through which a three-dimensional solid object, virtually of any shape, is generated starting from a digital model. Medical 3D printing was once an ambitious pipe dream. However, time and investment made it real. Nowadays, the 3D printing technology represents a big opportunity to help pharmaceutical and medical companies to create more specific drugs, enabling a rapid production of medical implants and changing the way that doctors and surgeons plan procedures [1]. This technology has multiple applications, and the fastest growing innovation in the medical field has been represented by the advent of the 3D printing itself [2]. Five technical steps are required to finalize a printed model. They include selecting the anatomical target area, the development of the 3D geometry through the processing of the medical images coming from a CT/MRI scan, the optimization of the file for the physical printing, and the appropriate selection of the 3D printer and materials (Figure 1). This file represents the guidance for the subsequent printing, “slicing” that digital design model into cross sections. That “sliced” design is then sent to a 3D printer, which manufactures the object by starting at the base layer and building a series of layers on top until the object is built using the raw materials that are needed for its composition. A patient-specific model with anatomical fidelity created from imaging dataset is finally obtained.

In this way, the 3D printing has the potential to significantly improve the research knowledge and the skills of the new generation of surgeons, the relationship between patient and surgeon [3], increasing the level of understanding of the disease involved, and the patient-specific design of implantable devices and surgical tools [4–6] and optimize the surgical process and cost [7]. Nowadays, different printing techniques and material are available in order to better reproduce the patient anatomy. Most of the available printing materials are rigid and therefore not optimum for flexibility and elasticity, unlike biological tissue [8]. Therefore, there are nowadays materials able to close the gap between the real anatomy and the reproduced one, especially considering the soft tissue [9, 10]. In this analysis, an overview of the 3D printing application in medical field is presented, highlighting the usefulness and limitations and how it could be useful for surgeons.

## 2. Additive Manufacturing Technologies

The 3D-printing techniques have grown in the last decades starting from 1986 when the first stereolithographic (SLA) systems were introduced in practice. Seven are the technical processes related to the 3D printing, each of which is represented by one or more commercial technologies, as shown by the ASTM International [11]. All the processes are listed in Table 1 that reported information about the technologies involved, the materials used, and the medical applications related to each process [12]. A comparison among all the seven techniques is proposed in the same table showing the advantages and disadvantages related to all the processes. Each process uses specific materials with specific properties that relate to medical applications, which are also summarized in Table 1. This general information helps the users to better choose the right technology depending on the application needed.

These technologies and the related advantages enable the researchers to improve existing medical applications that use 3D-printing technology and to explore new ones. The medical goal that has been already reached is significant and exciting, but some of the more revolutionary applications, such as bio/organ printing, require more time to evolve [2].

## 3. Transformation Process and Materials Used

Materials used in 3D printing are transformed during the production of the specific model by changing their consistency. This process is named cure and can be done in different ways: a melting of a hard filament in order to give the desired form to the model by the material distortion, liquid solidification for the construction of the structure and powder solidification. All these processes require filler or support material in lattice forms avoiding distortion of the model while the material is being cured. The support material can be easily removed by hand with a cutting tool; however, there is the risk to leave impression on the surface requiring an additional polishing in order to obtain a good-quality printing. The risk of damaging the model, losing details, or break the geometry is really high [23].

The correct selection of the material is directly linked to the selection of the 3D-printing process and printer, as well as the requirements of the model. Related to medical application, similarly to other applications, different anatomical structures need different mechanical properties of the materials to fulfill the required performance of the printed object [8]. The main distinction among the different materials that characterize the human body is between rigid and soft materials. Human bones are an example of rigid tissue and ligaments or articular cartilage are examples of soft materials. Bones are the simplest and easiest biological tissue to be produced by 3D printing as the majority of the materials are rigid. The materials used in 3D printing to model the bone structure are for example acrylonitrile butadiene styrene (ABS) [23], powder of plasters [24], and hydroquinone [8].

Relating to soft tissues, deeper research is still needed in order to decrease the gap between a 3D-printed anatomical model and the human structure. Most of the 3D-printing materials present a lack of realism to mimic adequately a soft human biological tissue. Thus, postprocessing may be necessary in order to soften the printed structures. Some examples are given in the reproduction of cartilaginous tissues [25], arteries for practicing valve replacement [26], hepatic segment [27], and hearts [28]. An interesting example is the development of a 3D-printed brain aneurysm using the flexible TangoPlus™ photopolymer [29] that represented a useful tool to plan the operative strategy in order to treat congenital heart disease. Furthermore, some of the materials used are urethane and rubber-like material, mixed with a rigid photopolymer, to reasonably mimic the artery structure due to their Shore value and elastic properties similar to the physiological one [30, 31].

For a promising future, the multimaterial composites seem to represent a good chance for the 3D printing of human tissues since none of the current available material is able to fully mimic elastic and biological tissues. Multimaterial composites may be designed based on the capacity of the selected biological material to replicate the mechanical properties of human tissue [32]. Mechanical testing may represent a necessary tool to analyze the biomechanical response and validate the artificial material.

Moreover, it is also important to mention that 3D printing allows the reproduction of implantable custom device, but still deeper research needs to be done in order to examine the differences between the traditional and additive manufacturing in terms of mechanical and structural properties, especially fatigue limit needs to be examined further [33].

## 4. Role of 3D Printing in Medical Field

Every year, 3D printing offers more and more applications in the healthcare field helping to save and improve lives in ways never imagined up to now. In fact, the 3D printing has been used in a wide range of healthcare settings including, but not limited to cardiothoracic surgery [34], cardiology [26], gastroenterology [35], neurosurgery [36], oral and maxillofacial surgery [37], ophthalmology [38], otolaryngology [39], orthopaedic surgery [22], plastic surgery [40], podiatry [41], pulmonology [42], radiation oncology [43], transplant surgery [44], urology [45], and vascular surgery [46].

Thanks to the different benefits that this technology could induce in the field, the main direct applications of 3D printing in the medical and clinical field are as follows [47]:

- Used for personalized presurgical/treatment and for preoperative planning. This will lead to a multistep procedure that, integrating clinical and imaging information, will determine the best therapeutic option. Several studies have demonstrated that patient-specific presurgical planning may potentially reduce time spent in the operating room (OR) and result in fewer complications [48, 49]. Moreover, this may lead to reduced postoperative stays, decreased reintervention rates, and lower healthcare costs. The 3D-printing technology allows to provide to the surgeon a physical 3D model of the desired patient anatomy that could be used to accurately plan the surgical approach along with cross-sectional imaging or, alternatively, modelling custom prosthetics (or surgical tool) based on patient-specific anatomy [50–54]. In this way, a better understanding of a complex anatomy unique to each case is allowed [52–56]. Furthermore, the 3D printing gives the possibility to choose before the implantation the size of the prostheses components with very high accuracy [57–59].
- Customize surgical tools and prostheses: the 3D printing can be used to manufacture custom implants or surgical guides and instruments. Therefore, the customization of surgical tools and prostheses means a reduction of cost given by the additive manufacturing technique [52–54, 60].
- Study of osteoporotic conditions: following a pharmacological treatment, 3D printing is useful in validating the results achieved by the patient. This enables a more accurate estimation of patientʼs bone condition and a better decision on the surgical treatment [15].
- Testing different device in specific pathways: a clear example is the reproduction of different vascular patterns to test the effectiveness of a cardiovascular system used to treat peripheral and coronary artery disease [61]. In this way, the 3D printing enables us to quickly produce prototypes of new design concepts or improvements to existing devices.
- Improving medical education: 3D-printed patient-specific models have demonstrated that they can increase performance and foster rapid learning [62], while significantly ameliorating the knowledge, management, and confidence of the trainees regardless of the area of expertise [8]. The benefits of 3D printing in education are the reproducibility and safety of the 3D-printed model with respect to the cadaver dissection, the possibility to model different physiologic and pathologic anatomy from a huge dataset of images, and the possibility to share 3D models among different institutions, especially with ones that have fewer resources [63]. 3D printers that have the capability to print with different densities and colours can be used to accentuate the anatomical details [64, 65].
- Patient education: patient-centered cares makes patient education one of the top priorities for most healthcare providers. However, communicating imaging reports verbally or by showing patients their CT or MRI scans may not be effective; the patients may not fully understand 2D images representation of a 3D anatomy. On the contrary, 3D printing may improve the doctor-patient communication by showing the anatomic model directly [66, 67].
- Storage of rare cases for educational purposes: this role is closely linked to the previous one. This allows the generation of a large dataset composed by datasets of patients affected by rare pathologies, allowing the training of surgeons in specific applications [52–54].
- Improve the forensic practice: in the courtroom, a 3D model could be used to easily demonstrate various anatomic abnormalities that may be difficult to jury members to understand using cross-sectional imaging [68].
- Bioprinting: the 3D printing allows also the modelling of implantable tissue. Some examples are the 3D printing of synthetic skin for transplanting to patients, who suffered burn injuries [69]. It may also be used for testing of cosmetic, chemical, and pharmaceutical products. Another example is the replicating of heart valves using a combination of cells and biomaterials to control the valve's stiffness [26] or the replicating of human ears using molds filled with a gel containing bovine cartilage cells suspended in collagen [70].
- Personalized drug 3D printing: the 3D printing of drugs consists of the printing out the powdered drug layer to make it dissolve faster than average pills [71]. It allows also personalization of the patient's needed quantity [2].
- Customizing synthetic organs: the 3D printing may represent an opportunity to save life reducing the waiting list of patients that need transplantation [72]. Bioprinted organs may also be used in the future by pharmaceutical industries to replace animal models for analyzing the toxicity of new drugs [73].

Therefore, these examples clearly demonstrated that 3D printing is one of the most disruptive technologies that have the potential to change significantly the clinical field, improving medicine and healthcare, making care affordable, accessible, and personalized. As printers evolve, printing biomaterials get safety regulated and the general public acquires a common sense about how 3D printing works.

### 4.1. Lack of Regulation

The biomedical field is one of the areas in which 3D printing has already shown its potentialities and that, in not too distant future, may be one of the key elements for the resolution of important problems related to human health that still exist.

Nowadays, despite the additive manufacturing offers a great potential for the manufacturing, the 3D-printing products do not have a proper legal status that defines them, both for implantable and nonimplantable devices. All the 3D-printed products are categorized as custom-made device under the Regulation (EU) 2017/745 of the European Parliament and of the Council of the 5 April 2017 [74]. They are defined as follow: “*any device specifically made in accordance with a written prescription of any person authorized by national law by virtue of that person's professional qualifications which gives, under that person's responsibility, specific design characteristics, and is intended for the sole use of a particular patient exclusively to meet their individual conditions and needs*”. Differently for mass-produced devices “*which need to be adapted to meet the specific requirements of any professional user and devices which are mass-produced by means of industrial manufacturing processes in accordance with the written prescriptions of any authorized person shall not be considered to be custom-made devices*” [75]. Indeed, manufacturers of custom-made devices shall only be guaranteed by an obligation of conformity assessment procedures upon which the device shall be compliant with safety and performance requirements [76]. Furthermore, the regulation states that “*Devices, other than custom-made or investigational devices, considered to be in conformity with the requirements of this Regulation shall bear the CE marking of conformity*” [77]. Thus, these medical devices do not require affixation of CE markings: a significant and constraining procedure demonstrating the safety and the performance of the device for the patient. Moreover, the custom-made devices do not require the UDI System (Unique Device Identification system) as reported in the Article 27, Comma 1 of the regulation.

A different approach has to be applied for custom-made implants, such as dental prostheses, that are defined as “*any device, including those that are partially or wholly absorbed, which is intended*:

- to be totally introduced into the human body, or
- to replace an epithelial surface or the surface of the eye,

*by clinical intervention and which is intended to remain in place after the procedure.*

*Any device intended to be partially introduced into the human body by clinical intervention and intended to remain in place after the procedure for at least 30 days shall also be deemed to be an implantable*.” [78]. The custom-made implantable devices require the CE marking in order to guarantee the safety and to be commercialized.

The EU has been working for many years on an update to the Medical Devices Directive. This proposed legislation has many noble attributes in addition to overcoming the gaps of the existing Medical Devices Directive, such as supporting technology and science innovation, while simultaneously strengthening patient safety. However, the current version of the draft Regulation lacks some depth that is mandatory to safeguard safe usage of 3D-printing technology and, thus, enable its increasing prevalence in medicine.

### 4.2. Examples of Application of 3D Printing in Paediatric Cases

Three-dimensional (3D) modelling and printing greatly supports advances in individualized medicine and surgery. Looking to the field of paediatrics, it is possible to identify four main applications categories: surgical planning, prostheses, tissue construct, and drug printing.

There are many successful cases that demonstrate the potential of the additive manufacturing in surgical planning in paediatric cases. In particular, most of the applications of 3D printing reported in the literature are related to the congenital heart disease [29]. This is due to the fact that children have a smaller chest cavity than adults, and the surgical treatment in paediatric cases may be much more difficult. The additive manufacturing helps the surgeons to have more information than the only ones that imaging technologies can afford. It helps the surgeon in the spatial orientation inside the cavities of a small infant heart and in simulating the surgical approach and steps of the operation with high fidelity [79]. This leads to shorter intraoperative time that per se has significant impact on complication rate, blood loss, postoperative length-of-stay, and reduced costs [80]. An example of the application of the 3D printing in the paediatric congenital heart disease treatment is a study reported in the literature based on the development of a 3D heart model of a 15-years-old boy to improve interventional simulation and planning in patient with aortic arch hypoplasia. The 3D-printed model allowed simulation of the stenting intervention. The assessment of optimal stent position, size, and length was found to be useful for the actual intervention in the patient. This represents one of the most technically challenging surgical procedures which opens the door for potential simulation applications of a 3D model in the field of catheterization and cardiovascular interventions [81].

Another study proposed in which the 3D printing had a relevant role consists in a clinical preoperative evaluation on five patients ranged from 7 months to 11 years of age affected by a double outlet right ventricle with two well-developed ventricles and with a remote ventricular septal defect. The three-dimensional printed model based on the data derived from computed tomography (CT) or magnetic resonance (MRI) contributed to a more complete appreciation of the intracardic anatomy, leading to a successful surgical repair for three of the five patients. [82] Lastly, CT and MRI data were used to construct 3D digital and anatomical models to plan a heart transplantation surgical procedure of two patients of 2 and 14 years old affected relatively by hypoplastic left heart syndrome and pulmonary atresia with a hypoplastic right ventricle. These physical models allowed the surgeon and the paediatric cardiologist to develop the optimal surgical treatment during the heart transplantation anticipating problems that may arise during the procedure. The specific dimensions and distances can be measured, and heart transplantation can be planned [83].

The importance of three-dimensional printing has been demonstrating also in other application. The additive manufacturing in fact has been used to plan surgical treatment of paediatric orthopaedic disorders [84]. The 3D model of a 2-year-old male child was produced in order to plan the surgical treatment for his multisutural craniosynostosis with a history of worsening cranial deformity. Other than the turribrachycephalic skull, the child also had greatly raised intracranial pressure with papilledema and copper beaten appearance of the skull. Thorough preoperative planning enabled faster surgery and decreased anesthesia time in a compromised patient [85].

Another study, based on 13 cases of multiplane spinal or pelvic deformity, was developed in order to demonstrate that the three-dimensional printing may represent a useful tool in the surgical planning of complex paediatric spinal deformities treatment [86].

Changing the final goal of the additive manufacturing, other applications cases are reported in the literature to demonstrate the usefulness in the production of paediatric patient-specific prostheses. An example in the literature is given by the development of a low-cost three-dimensional printed prosthetic hand for children with upper-limb reductions using a fitting methodology that can be performed at a distance [87]. This specific case demonstrates that the advancements in computer-aided design (CAD) programs, additive manufacturing, and imaging editing software offer the possibility of designing, printing, and fitting prosthetic hands devices overcoming the costs limitation. As a consequence, the advantages of 3D-printed implants over conventional ones are in terms of customizability and cost as seems to be clear from the previous example. On the contrary, the major adversity is related to the rapid physical growth that makes the customize prostheses outsized frequently. This leads to the production of advanced technological implant that, due to their high complexity and weight, increases cost. The additive manufacturing can be used to fabricate rugged, light-weight, easily replaceable, and very low-cost prostheses for children [88]. The major prostheses lack is related to the ability to communicate with the brain in terms of sensibility. With the advent of bioprinting, cellular prostheses could be an interesting area of research, which can lead to integrated prostheses in the brain communication system, and exhibit more biomimicry with tissue and organ functionalities [89].

Related to bioprinting, there are few applications nowadays involved in the tissues production in regenerative medicine. Many different tissues have been successfully bioprinted as reported in many journal articles [90] including bone, cartilage, skin, and even heart valves. However, the bioprinted tissues and organs are at the laboratory level; a long way needs to be travelled to achieve successful clinical application [91].

Last but not the least, the additive manufacturing in terms of drug printing may also represent an innovative technique in the production of patient-specific medicine with regard to the composition and the dose needed by the patients. The drug-printing introduces the concept of tailor-made drugs in order to make drugs safer and more effective. Especially for children, furthermore, drug-printing represents the possibility of choosing colour, shape, and design of the medication, reducing the resistance in taking them. Imagine a paediatrician talking to a four-year-old child who is having trouble adjusting to taking daily doses of steroids after being diagnosed with Duchenne muscular dystrophy the previous month. 3D printing allows us to design in particular shape the drug, making medicine more appealing to the child [92]. It is amental to note that changing the shape of a capsule does not have to lead to different dose and drug properties, such as drug release or dissolution rate [93].

## 5. Conclusions

The 3D printing in medical field and design needs to think outside the norm for changing the health care. The three main pillars of this new technology are the ability to treat more people where it previously was not feasible, to obtain outcomes for patients and less time required under the direct case of medical specialists. In few words, 3D printing consists in “enabling doctors to treat more patients, without sacrificing results” [94].

Therefore, like any new technology, 3D printing has introduced many advantages and possibilities in the medical field. Each specific case in which 3D printing has found application shown in this analysis is a demonstration of this. However, it must be accompanied by an updated and current legislation in order to guarantee its correct use.

## Figures and Tables

**Figure 1:** 3D-printing workflow.

**Table 1:** Summary of the 3D-printing process and technologies, focus on materials needed and medical applications, and comparison among the 3D-printing technologies.

Designation additive-manufacturing process	Process description	Technologies	Materials	Medical use	Pros	Cons
Vat photo-polymerisation	Vat polymerisation uses a vat of liquid photopolymer resin, out of which the model is constructed layer by layer	Stereolithography (SLA) Digital light processing (DLP)	(i) Photopolymer resin	Bone, dental models [13], dental implant guides [14], hearing aids [15]	(i) High resolution and accuracy (ii) Complex parts (iii) Decent surface finish: smoother finish (iv) Flexible printing setup	(i) Lacking in strength and durability (ii) Still affected by UV light after print (iii) Not for heavy use

Material jetting	Material jetting creates objects in a similar method to a two-dimensional ink jet printer. Material is jetted onto a build platform using either a continuous or drop on demand (DOD) approach	Multijet modelling (MJM)	(i) Plastics (ii) Polymers: polypropylene, HDPE, PS, PMMA, PC, ABS, HIPS, EDP	Medical models [16], dental casts, dental implant guides [17]	(i) High accuracy (ii) Low waste of material (iii) Multiple material parts and colours in one process	(i) Required support material (ii) Limited materials: only polymers and waxes are supported

Binder jetting	The binder-jetting process uses two materials; a powder-based material and a binder. The binder is usually in liquid form and the build material in powder form. A print head moves horizontally along the *x* and *y* axes of the machine and deposits alternating layers of the build material and the binding material	Powder bed and inkjet head 3D printing (PDIH) Plaster-based 3D printing (PP)	(i) Stainless steel (ii) Polymers: ABS, PA, PC (iii) Ceramics: glass	Colour models especially colour coding of anatomy [18]	(i) Range of colours (ii) Multiple materials supported (iii) Faster (iv) Different binder-powder combination for various mechanical properties	(i) Not always suitable for structural parts (ii) The cleaning of the 3D-printing result needs time and increases the time of the procedure

Material extrusion	Fuse deposition modelling (FDM) is a common material extrusion process and is trademarked by the company Stratasys. Material is drawn through a nozzle, where it is heated and is then deposited layer by layer. The nozzle can move horizontally, and a platform moves up and down vertically after each new layer is deposited	Fused deposition modelling (FDM) Fused filament fabrication (FFF)	(i) Plastics; (ii) Polymers: ABS, nylon, PC, AB	Medical instruments and devices [19], rapid prototyping exoskeleton [20]	(i) Inexpensive process (ii) Widespread (iii) ABS plastic supported: good structural properties and easily accessible	(i) Dependence of quality on the noozle radius: bigger nozzle leads to less quality (ii) Low accuracy and dependence on the nozzle thickness (iii) Low speed (iv) Contact pressure needed to increase quality
Powder bed fusion	The powder bed fusion process includes the following commonly used printing techniques: direct metal laser sintering (DMLS), electron beam melting (EBM), selective heat sintering (SHS), selective laser melting (SLM) and selective laser sintering (SLS)	Selective laser sintering (SLS) Direct metal laser sintering (DMLS) Selective heat sintering (SHS) Selective laser melting (SLM) Electron beam melting (EBM)	Powder-based materials. Common metals and polymers used are (i) SHS: nylon (ii) DMLS, SLS, SLM: stainless steel, titanium, aluminium, cobalt chrome, steel (iii) EBM: titanium, cobalt chrome, stainless steel material, aluminium and copper	Models that require a lattice, medical devices such as implants and fixations [21]	(i) Inexpensive (ii) Small technology: office size machine (iii) Large range of material options	(i) Low speed; lack of structural properties in materials (ii) Limited sizes (iii) Dependence on powder grain size

Sheet lamination	Sheet lamination processes include ultrasonic additive manufacturing (UAM) and laminated object manufacturing (LOM). The ultrasonic additive manufacturing process uses sheets or ribbons of metal, which are bound together using ultrasonic welding	Laminated object manufacturing (LOM) Ultrasonic consolidation (UC)	Paper, plastic and sheet metals	Orthopaedic modelling of bone surfaces [22]	(i) Speed (ii) Inexpensive (iii) Ease of materials handling	(i) Dependence on paper or plastic material (ii) Need of postprocessing (iii) Limited material range

Direct energy deposition	Directed energy deposition (DED) covers a range of terminology: “Laser engineered net shaping, directed light fabrication, direct metal deposition, 3D laser cladding” it is a more complex printing process commonly used to repair or add additional material to existing components	Laser metal deposition (LMD)	Metals: cobalt chrome, titanium	Limited. Commonly used to repair existing parts and build very large parts	(i) High control of grain structure (ii) High-quality-dependent on speed (iii) High-accuracy-dependent on accuracy (iv) Fast built with rapid material deposition (v) Fully dense parts; no need for supports (vi) Best process for part repair	(i) Limited range of materials; (ii) Poor surface quality; (iii) Wire process is less accurate
